# Mathematical Simulation and Numerical Computation of the Temperature Profiles in the Peripherals of Human Brain during the Tepid Sponge Treatment to Fever

**DOI:** 10.1155/2022/2658095

**Published:** 2022-01-17

**Authors:** Mir Aijaz, Javid Gani Dar, Ibrahim M. Almanjahie, Irsa Sajjad

**Affiliations:** ^1^Department of Mathematics, Govt. Degree College Kilam, Higher Education, J & K, India; ^2^Department of Mathematical Sciences, Islamic University of Science and Technology, J & K, India; ^3^Department of Mathematics, College of Science, King Khalid University, Abha 62529, Saudi Arabia; ^4^Statistical Research and Studies Unit, King Khalid University, Abha 62529, Saudi Arabia; ^5^Department of Business Sciences, Ibadat International University, Islamabad, Pakistan

## Abstract

**Background:**

Fever is one of the frequently occurring diseases in human beings, and the body is said to have befallen in fever if the arterial or internal body temperature rises to 38°C. The patient who suffers from fever is either given paracetamol or tepid sponging or both.

**Objective:**

This paper is aimed at studying the effects of the tepid sponge in normalizing the high temperature of the human body during fever. Among the various available methods for tepid sponging, the impact of holding a cool wet cloth on the forehead for reducing the fever is analyzed and pictured graphically.

**Method:**

For analyzing the effects of tepid sponge on the temperature distribution of the domain consisting of scalp, skull, and cerebrospinal fluid (CSF), a cool wet cloth is brought in contact with the skin allowing the heat to transfer from the brain to the wet cloth through these layers. The heat transfer in living biological tissues is different from ordinary heat transfer in other nonliving materials. Therefore, a model based on the bioheat equation has been constructed. The model has been solved by numerical methods for both steady- and unsteady-state cases. The domain, which consists of the scalp, skull, and CSF layers of the human head, has been discretized into four equal parts along the axes of the three-dimensional coordinate system. The forward difference and forward time centered space approximations were employed for numerical temperature distribution results at the nodal points.

**Results:**

The effects of tepid sponge in reducing the body temperature with fever at 38°C, 39.5°C, and 41°C have been numerically calculated, and the results were pictured graphically. For transient cases, the corresponding calculations have been carried out at times *t* = 2 minutes, 4 minutes, and 6 minutes.

**Conclusion:**

Among all the available remedies to fever, tepid sponging has shown a significant effect in controlling fever.

## 1. Introduction

Fever is one of the common and universally known diseases from which human beings frequently suffer. Fever is generally the body's response to infection [1]. Fever is said to occur when the oral temperature exceeds 38°C. The normal range of oral temperature of the human body is 37.2–37.7°C as asserted by Mackowiak et al. [2]. The findings of Mackowiak et al. [2] conflicted with Wunderlich's definition of the normal temperature of the human body as the latter had ranged it between 36.8 and 37°C. The authors exhibited comparable thermal variability and observed experimentally that the mean oral temperature of our body varies with the time of day (morning, noon, or evening) and sex (men or women). Morrison et al. [3] demonstrated that the central neural circuits orchestrate a homeostatic repertoire to maintain the body temperature during abnormal environmental conditions and to alter body temperature during the inflammatory response.

Man has always been striving for remedies to various diseases and has been experimenting with drug placebo and physical methods for optimum outcomes. Treatment of fever by tepid sponging at home, especially to children by caregivers prior to a doctor's consultation, is a common practice, and it changes the temperature of the body significantly, as analyzed by Hendrawati and Elvira [4]. Tepid or cold sponging is a remedy where the application of moist cold liquid reduces the excess temperature of the body. Although, this treatment at home is generally successful but sometimes may lead to complications due to mishandling by a person with negligible medical competency. The treatment techniques employed include exposing the patient to air, tepid sponging, and using drugs such as paracetamol and other traditional remedies [5]. Among all these treatments, tepid sponging is most commonly practiced. The sponging action is a process where the water film by cool wet cloth is constantly pressed and moved over a part of the body, especially the forehead, resulting in the replacement of the warm water with a fresh layer of cooler water on the skin surface, thus helping in maximizing the outward heat transfer through conduction, convection, and perfusion [6].

Aluka et al. [7] compared the treatment by cold water sponging with paracetamol on children and analyzed the effects of both for the reduction of fever temperature. They substantiated that as compared to oral paracetamol, cold water sponging yields a more speedy reduction in body temperature of febrile children in a tropical environment, and the results are more effective when the sponging is ongoing. Meremikwu et al. [8] also observed the effect of physical methods versus drug placebo or no treatment for managing fever in children. Further, the comparisons of the various treatments like alcohol versus tepid sponging, iced water versus tepid sponging, and physical methods versus drug injection were carried and analyzed. Agbolosu et al. [9] studied the efficacy of tepid sponging over paracetamol on a sample of 80 children, among which 40 were enrolled for paracetamol treatment and the remaining 40 for tepid sponging. They concluded that in a tropical climate, paracetamol is more effective in reducing fever than tepid sponging. However, tepid sponging together with paracetamol is highly effective in serving the purpose of reducing the patient's excess temperature due to fever. Eman [10] considered the problem of heat transfer in the skin tissue of the human head subjected to thermal diffusion with relaxation time and concluded that the values of the time and the distance have significant effects on the temperature increment and temperature concentration. The values of the temperature increment and the concentration increase when the time increases, and their values decrease when the distance increases. Shen et al. [11] examined the heat transfer and elastic deformation in soft tissues by using Penne's bioheat transfer equation and the modified Duhamel-Neumann equations. A 19-point finite-difference scheme was used to solve the three-dimensional governing equation. Ferreira and Yanagihara [12] also solved the model based on 3D heat conduction and used the elliptical cylinders to adequately approximate the body geometry.

The present paper explores the three-dimensional heat transfer and corresponding temperature distribution during tepid sponging treatment to fever. The water, being a compound with high specific heat capacity, is an excellent and readily available material for extracting the heat from the patient's body. Thus, when a piece of wet cloth is kept on the forehead, it immediately cools down the temperature of the scalp and hence of the skull and CSF. This paper derives a mathematical estimation of temperature distribution in the scalp, skull, and CSF (the surrounding layers of the human brain) during tepid sponging treatment in fever. The temperature of the skin decreases due to its contact with a piece of wet cloth which is repeatedly damped in cold water, wrung for any extra moisture, and applied to the forehead. The heat (due to fever) from the body is taken away by the water resulting in cooling down the temperature of the forehead and, in turn, reducing the fever in subsequent regions. Aijaz et al. [13] elaborated how the water that diffuses into the skin plays a significant role in the fluctuation of temperature profiles near the skin surface and subsequent regions. Khanday et al. [14] estimated the fluid distribution patterns in human skin at various values of metabolic heat generation. Further, Tsunetsugu and Sugiyama [15] compared the physiological changes in the human body which is in direct contact with various materials especially wood. In a similar way, during tepid sponging treatment, the skin is in direct contact with wet cloth; therefore, heat flows out through biological tissues involving conduction, convection, and perfusion processes. Further, various physiological parameters have a remarkable impact on the heat transfer through tissue as assessed by Ley and Bayazitoglu [16]. Therefore, for the formulation of the mathematical model, Pennes' bioheat equation [17] is the most appropriate equation as discussed by Aijaz et al. [18]. Therefore, the rate of heat flow through the human head is also dependent on the layer under study. Hence, for better results, it becomes imperative to discretize the domain into small elements. In this direction, the model has been solved for both steady- and unsteady-state cases by the forward difference approximation and the forward time centered space (FTCS), respectively. The uniform grid of dimensions *h* × *h* × *h* is introduced, and then, the differential equations for internal node (*x*_*i*_, *y*_*j*_, *z*_*k*_) have been solved as demonstrated by Majchrzak and Turchan [19].

## 2. Materials and Methods

We intend to formulate a model for estimating the heat transfer in the domain consisting of scalp, skull, and CSF during tepid sponging. Therefore, to make the domain compatible with the three-dimensional coordinate system, we take both a piece of wet cloth and the part of the forehead which is in contact with it as cuboidal shaped. Let the domain be of length *L* = *l*_1_ (along the +ve *x*-axis), height *H* = *l*_2_ − *l*_5_ (along the *y*-axis), and width *W* = *l*_3_ − *l*_4_ (along the *z*-axis). *l*_2_, *l*_3_, *l*_4_, and *l*_5_ are five points on the surface of wet cloth equidistant from the origin as shown in Figure 1(a), and *l*_1_ is the extreme point (the interface between CSF and brain) up to which heat transfer is to be estimated. The diffusion equation applicable to the present in vivo heat transfer is the three-dimensional bioheat equation given by

(1) $$\begin{array}{c} \rho c\frac{\partial T}{\partial t}=\frac{\partial }{\partial x}\left(k\frac{\partial T}{\partial x}\right)+\frac{\partial }{\partial y}\left(k\frac{\partial T}{\partial y}\right)+\frac{\partial }{\partial z}\left(k\frac{\partial T}{\partial z}\right)+m_{b}c_{b}\left(T_{A}-T\right)+Q_{m}+Q_{e}, \end{array}$$

where *T*, *k*, *ρ*, and *c* are, respectively, the temperature, the thermal conductivity, the density, and the specific heat capacity of the tissue. *m*_*b*_ is the blood perfusion rate, *c*_*b*_ is the specific heat of the blood, and *T*_*A*_ is the arterial blood temperature, but in the present paper, it is fever temperature which is 38°C, 39.5°C, and 41°C for three different cases. *Q*_*m*_ and *Q*_*e*_ are, respectively, the metabolic heat generation and effect by external cooling source. In this paper, the external cooling source is the wet cloth used for tepid sponging at a uniform temperature of 7°C.

It is to be noted that *k*, *p*, and *c* have specific constant values in each layer of the domain and, hence, take distinct values in scalp, skull, and CSF as demonstrated by Aijaz et al. [18]. Thus, in the numerical computation, their numerical values will be taken according to the positions of nodal points pertaining to *T*_*i*,*j*,*k*_ in the numerical discretization of the domain (see Figure 1(b)). The appropriate boundary conditions for Equation (1) are

(2) $$\begin{array}{c} \left\{\begin{array}{c} k\frac{\partial T}{\partial x}=h_{e}\left(T-T_{w}\right)\text{ at }x=0,\\ k\frac{\partial T}{\partial y}=0\text{ at }y=l_{2},l_{5},\\ k\frac{\partial T}{\partial z}=0\text{ at }z=l_{3},l_{4}, \end{array}\right. \end{array}$$

where *h*_*e*_ is the heat transfer coefficient and *T*_*w*_ is the temperature of the wet cloth. (*l*_1_ − 0) × (*l*_2_ − *l*_5_) × (*l*_4_ − *l*_3_) are the dimensions of the body part which is beneath tepid sponging and (*l*_2_ − *l*_5_) × (*l*_4_ − *l*_3_) is the surface area of the skin under tepid sponging.

In the biological system of human beings, the heat not only transfers through conduction but also by perfusion through blood circulation; see, for example, Aijaz et al. [20]. Further, the heat transfer in humans also depends upon the metabolic heat generation and the impact of the external heat source as well as ambient temperature. The heat loss due to tepid sponging of the fevered body involves the heat transfer through human tissue; therefore, the bioheat equation is the most appropriate equation for the formulation of the model. The cubical domain of the model is discretized into small elements having meshes and nodes. This paper studies the effects of a tepid sponge on a small cuboidal portion of the forehead of the human body. Therefore, this assumption does not depart the model from the actual situation. The values of the temperature at the nodes on the boundary of the domain are known. To get the needed results and make the numerical calculations simple, finite difference methods (forward/backward/central difference approximations) are the most appropriate methods. However, in this paper, we shall opt for the forward difference method as it is frequently used in numerical methods and hence simple. For more generalized results, Equation (1) can be solved for both steady-state case and transient case.

## 3. Steady-State Case

The steady-state case of Equation (1) reduces to

(3) $$\begin{array}{c} k\left\{\frac{\partial^{2}T}{\partial x^{2}}+\frac{\partial^{2}T}{\partial y^{2}}+\frac{\partial^{2}T}{\partial z^{2}}\right\}-m_{b}c_{b}T=-\left(m_{b}c_{b}T_{A}+Q_{m}+Q_{e}\right). \end{array}$$

For numerical approximations, the unit of discretization along all the axes is the same and is denoted by *h* (numerically equal to 2 mm). So, the domain discretizes into 64 small cubes each of size 2 mm × 2 mm × 2 mm, as shown in Figure 2. Thus, the forward difference approximation at the point (*ih*, *jh*, *kh*) is

(4) $$\begin{array}{c} k\left\{\frac{T_{i-1,j,k}-2T_{i,j,k}+T_{i+1,j,k}}{h^{2}}+\frac{T_{i,j-1,k}-2T_{i,j,k}+T_{i,j+1,k}}{h^{2}}+\frac{T_{i,j,k-1}-2T_{i,j,k}+T_{i,j,k+1}}{h^{2}}\right\}-m_{b}c_{b}T_{i,j,k}=-\left(m_{b}c_{b}T_{A}+Q_{m}+Q_{e}\right)\Rightarrow T_{i-1,j,k}+T_{i+1,j,k}+T_{i,j-1,k}+T_{i,j+1,k}+T_{i,j,k-1}+T_{i,j,k+1}-\left(6+\frac{h^{2}}{k}m_{b}c_{b}\right)T_{i,j,k}=-\frac{h^{2}}{k}\left(m_{b}c_{b}T_{A}+Q_{m}+Q_{e}\right). \end{array}$$

The outer skin is in touch with the wet cloth. Therefore, the heat transfer coefficient is incorporated at the outer layer of the skin. We consider the cuboidal domain; hence, the temperature gradient at the five boundaries (excluding *yz* plane, i.e., where *x* = 0) can be taken as zero. Thus, the boundary conditions are

(5) $$\begin{array}{c} \left.\begin{array}{c} k\frac{\partial T}{\partial x}=h_{e}\left(T-T_{w}\right)\;\text{at}\;x=0,\;k\frac{\partial T}{\partial x}=0\;\text{at}\;x=l_{1}\\ k\frac{\partial T}{\partial y}=0\;\text{at}\;y=l_{2},l_{5}\;k\frac{\partial T}{\partial z}=0\;\text{at}\;z=l_{3},l_{4} \end{array}\right\}. \end{array}$$

Further, assuming that the wet cloth is dipped in cold water making the temperature of cloth 7°C uniformly, i.e., *T*_*i*,*j*,*k*_ = 7.0°C for *i* = 0; *j*, *k* = 0, ±1; ±2. Fever is generally said to occur when the internal body temperature exceeds 38°C. Therefore, we take the situations when the internal body temperature due to fever is 38°C, 39.5°C, and 41°C for the three different cases as shown in Tables 1–3, respectively, where

(6) $$\begin{array}{c} \left.\begin{array}{cc} T_{A} & =38.0^{\circ }\text{C for }i=5;j,k=0,\pm 1;\pm 2\;\left(\text{Case I}\right)\\ \; & =39.5^{\circ }\text{C for }i=5;j,k=0,\pm 1;\pm 2\;\left(\text{Case II}\right)\\ \; & =41.0^{\circ }\text{C for }i=5;j,k=0,\pm 1;\pm 2\;\left(\text{Case III}\right) \end{array}\right\}. \end{array}$$

Discretizing the domain into four subintervals along the *x*-axis, resulting in three unknown points on the *x*-axis, so that, for three-dimensional discretization, there are 3 × 3 × 3 = 27 unknown points. Giving *i* = 1, 2, 3; *j* = 1, 2, 3; *k* = 1, 2, 3 in (4), we obtain 27 linear equations for 27 points of *T*_*i*,*j*,*k*_ with matrix form of these equations as

(7) $$\begin{array}{c} M_{27\times 27}T_{27\times 1}=N_{27\times 1},\\ \Rightarrow T=M^{-1}N, \end{array}$$

where

(8) $$\begin{array}{c} M=\left(\begin{array}{cccccc} -\left(6+h^{2}a_{1}\right) & 1 & 0 & \cdots & 0 & 0\\ 1 & -\left(6+h^{2}a_{2}\right) & 1 & \cdots & 0 & 0\\ 0 & 1 & -\left(6+h^{2}a_{3}\right) & \cdots & 0 & 0\\ \cdots & \cdots & \cdots & \cdots & \cdots & \cdots \\ \cdots & \cdots & \cdots & \cdots & \cdots & \cdots \\ 0 & 0 & 0 & \cdots & -\left(6+h^{2}a_{26}\right) & 1\\ 0 & 0 & 0 & \cdots & 1 & -\left(6+h^{2}a_{27}\right) \end{array}\right),\\ T=\left(\begin{array}{c} T_{1,1,1}\\ T_{1,1,2}\\ T_{1,1,3}\\ \cdots \\ T_{3,3,2}\\ T_{3,3,3} \end{array}\right),\\ N=\left(\begin{array}{c} -h^{2}b_{1}\\ -h^{2}b_{2}\\ -h^{2}b_{3}\\ \cdots \\ -h^{2}b_{26}\\ -h^{2}b_{27} \end{array}\right). \end{array}$$

The constants *a*_*i*_ and *b*_*i*_, *i* = 1, 2, 3 ⋯ 27, are defined as

(9) $$\begin{array}{c} \left.\begin{array}{cc} a_{i} & =\frac{h^{2}}{k_{e}}m_{b}c_{b}\text{ if }T_{i,j,k}\text{ falls in the subdomain scalp}\\ \; & =\frac{h^{2}}{k_{d}}m_{b}c_{b}\text{ if }T_{i,j,k}\text{ falls in the subdomain skull}\\ \; & =\frac{h^{2}}{k_{h}}m_{b}c_{b}\text{ if }T_{i,j,k}\text{ falls in the subdomain CSF} \end{array}\right\},\\ \left.\begin{array}{cc} b_{i} & =-\frac{h^{2}}{k_{e}}\left\{m_{b}c_{b}+{\left(Q_{m}\right)}_{e}+Q_{e}\right\}\text{ if }T_{i,j,k}\text{ falls in the subdomain scalp}\\ \; & =-\frac{h^{2}}{k_{d}}\left\{m_{b}c_{b}+{\left(Q_{m}\right)}_{d}+Q_{e}\right\}\text{ if }T_{i,j,k}\text{ falls in the skull}\\ \; & =-\frac{h^{2}}{k_{h}}\left\{m_{b}c_{b}+{\left(Q_{m}\right)}_{h}+Q_{e}\right\}\text{ if }T_{i,j,k}\text{ falls in the subdomain CSF} \end{array}\right\}. \end{array}$$

MATLAB software has been used for the numerical solutions of *T*_*i*,*j*,*k*_. Then, for more accurate values, the domain discretization has been refined and numerical values have been enlisted in Tables 1–3 and displayed in Figures 3–5.

## 4. Transient Case

The corresponding numerical approximation of Equation (1) is based on the forward difference approximation for the time derivative and centered difference approximation for the space derivatives applied at the point (*ih*, *jh*, *kh*, *nd*). Thus, by FTCS (forward time centered space) method, we have

(10) $$\begin{array}{c} \rho c\frac{T_{i,j,k}^{n+1}-T_{i,j,k}^{n}}{d}=k\left(\frac{T_{i-1,j,k}^{n}-2T_{i,j,k}^{n}+T_{i+1,j,k}^{n}}{h^{2}}+\frac{T_{i,j-1,k}^{n}-2T_{i,j,k}^{n}+T_{i,j+1,k}^{n}}{h^{2}}+\frac{T_{i,j,k-1}^{n}-2T_{i,j,k}^{n}+T_{i,j,k+1}^{n}}{h^{2}}\right)+m_{b}c_{b}T_{A}-m_{b}c_{b}T_{i,j,k}^{n}+Q_{m}+Q_{e}\Rightarrow T_{i,j,k}^{n+1}=\frac{dk}{h^{2}\rho c}\left\{\left(T_{i-1,j,k}^{n}-T_{i+1,j,k}^{n}\right)+\left(T_{i,j-1,k}^{n}-T_{i,j+1,k}^{n}\right)+\left(T_{i,j,k-1}^{n}-T_{i,j,k+1}^{n}\right)\right\}+\left(\frac{6kd}{h^{2}\rho c}+\frac{d}{\rho c}m_{b}c_{b}+1\right)T_{i,j+1,k}^{n}+\frac{d}{\rho c}\left(Q_{m}+Q_{e}\right), \end{array}$$

where *h* (numerically equal to 2 mm) is the uniform length of elements between two adjacent nodes and *d* (numerically equal to 2 minutes) is the time interval between two consecutive readings.

The boundary conditions are the same as discussed in the steady-state case (5), and the initial conditions are

(11) $$\begin{array}{c} T_{i,j,k}^{n}=7^{\circ }C\text{ for }n=0,i=0,j,k=0,\pm 1,\pm 2=T_{A}\text{ for }n=0,i=4,j,k=0,\pm 1,\pm 2. \end{array}$$

Furthermore, the various values of fever temperature *T*_*A*_ for the transient case are the same as given by (6). The temperature of the surface of wet cloth covering the skin of the forehead is reset to 7°C after a time interval of 2 minutes, and the results are recomputed for numerical approximations of the temperature profiles as shown in Tables 4–6.

## 5. Domain Discretization and Numerical Scheme

The domain considered for tepid sponging is of the cuboidal shape having its outer skin surface as *yz* plane, and the *x*-axis is in the normal direction to the skin surface. Excluding boundaries, three equidistant points *x*_1_, *x*_2_, and *x*_3_ are taken along the *x*-axis in the domain. Similarly, take the equally spaced points *y*_1_, *y*_2_, and *y*_3_ along the *y*-axis and *z*_1_, *z*_2_, and *z*_3_ along the *z*-axis inside the cuboidal domain as shown in Figure 2. For austerity, the three-dimensional frame is chosen in such a way that the point (*x*_0_, *y*_2_, *z*_2_) represents origin, i.e., *x*_0_ = *y*_2_ = *z*_2_ = 0. The domain so formed has known values of temperatures at peripheral boundaries. The forward difference approximation (in steady-state case) and forward time centered space (in transient case) are employed to find the numerical values of the temperatures at the different mesh points of the gridded domain. The discretization of the domain is based on the variation of numerical values of the physiological parameters of the forehead as elucidated by Ley and Bayazitoglu [16].

## 6. Results and Discussions

A mathematical model based on the bioheat equation has been formulated to study the temperature distribution and heat transfer in the scalp, skull, and CSF of the forehead during tepid sponging treatment to fever. The bioheat equation is preferred because it incorporates those parameters which make a significant contribution to heat transfer. The model has been solved for the numerical results by the forward difference method for the steady-state case and by the forward time centered space for the transient case separately. To display the results graphically, it becomes indispensable to get the numerical approximations by using the numerical values of the parameters. The numerical values of all the associated parameters (see Table 7) have been taken from the various research papers which include Khanday et al. [14], Janssen et al. [21], Aijaz et al. [18], Shirkavand and Nazif [22], Melo et al. [23], de Dear et al. [24], and Giering et al. [25]. It is to be noted that there is a small variation in the values of the thickness of scalp, skull, and CSF, depending on the age and geographical factors. In this model, we shall take the average thickness of these layers as scalp = 4.5 mm, skull = 3.5 mm, and CSF = 2 mm.

Temperature distribution in the domain which lies under the wet cloth during tepid sponging is computed numerically. The temperature distribution for the steady-state case is shown in Table 1 (at fever 38°C), Table 2 (at fever 39.5°C), and Table 3 (at fever 41°C). For the transient case, the temperature distribution in the domain has been computed at *t* = 2 min, 4 min, and 6 min as shown in Table 4 (at fever 38°C), Table 5 (at fever 39.5°C), and Table 6 (at fever 41°C). These results have also been displayed graphically in Figures 3–5 (steady-state case) and Figures 6–8 (transient case).

In Figure 9, a comparison of the temperature distribution obtained before and after tepid sponging treatment in the patient's forehead has been pictured.  Figure 10 shows the comparison of the temperature distribution, recorded before and after tepid sponging at *t* = 2 minutes, *t* = 4 minutes, and *t* = 6 minutes. Based on the results obtained for the heat transfer and the temperature distribution during tepid sponging, it is evident from the tables and graphs that tepid sponging has shown a positive effect on the reduction of fever. The fevered body temperature regulates to normal temperature in a few minutes giving the patient relief and comfort.

## 7. Conclusion

Tepid sponging is one of the old practices used for the treatment of fever. Just at the beginning of the tepid sponging, the fever at the outer surface seems to have been normalized, but the internal parts of the body and the exterior layers of the brain are still in fever. Therefore, for diagnosing the effects of tepid sponging treatment for reducing temperature due to fever, continuous monitoring of temperature distribution needs to be tracked by some means. The various processes like temperature regulation and mechanism of fever control are also playing their part in reducing fever. In the present paper, an effort has been made to show the temperature variation numerically in the various layers of the forehead during tepid sponging. Therefore, the present paper can be a good tool in analyzing the significance of tepid sponging treatment for fever. Hence, or otherwise, a combination therapy (tepid sponging and paracetamol) could be effective in the treatment of fever. From Figures 3–8, it can be concluded that the reduction of temperature due to tepid sponging at outer surface drops quickly and the process of heat transfer starts for the rest of the layers of the domain. Moreover, Figures 9 and 10 show a blueprint picture of the comparison (before and after tepid sponging) of the temperature distribution in the domain.

Among the various treatments for fever, tepid sponging is useful, result-oriented, readily available, and without side effects. Generally, tepid sponging works nicely for some time, and then, it needs to be combined with paracetamol. The present study helps in determining whether the treatment by the tepid sponge is sufficient or not. If not, after how much time, tepid sponging is to be discontinued or supplemented with paracetamol. The diffusion of fluids and the heat transfer through the skin (and hence the other regions under it) of the forehead is different from the skin at the other parts of the human body as estimated by Eman [10]. Therefore, the results cannot be directly applied to other parts of the body. However, there is a scope for improving this paper for the other parts of the human body. The novelty of this paper over the experimental-based papers is that the needed results can be directly obtained from this model by giving the numerical values to the parameter used in the formulation of the model.

## Figures and Tables

**Figure 1:** (a) Domain of the model as (*l*_1_ − 0) × (*l*_2_ − *l*_5_) × (*l*_4_ − *l*_3_). (b) 3D representation of a point in the domain.

**Figure 2:** Discretization of the domain in 3D coordinate system.

**Figure 3:** Temperature distribution in the domain after tepid sponge treatment with initial fever or arterial temperature *T*_*A*_ = 38.0°C (steady-state case).

**Figure 4:** Temperature distribution in the domain after tepid sponge treatment with initial fever or arterial temperature *T*_*A*_ = 39.5°C (steady-state case).

**Figure 5:** Temperature distribution in the domain after tepid sponge treatment with initial fever or arterial temperature *T*_*A*_ = 41.0°C (steady-state case).

**Figure 6:** Temperature distribution in the domain after tepid sponge treatment with initial fever or arterial temperature *T*_*A*_ = 38.0°C (transient case).

**Figure 7:** Temperature distribution in the domain after tepid sponge treatment with initial fever or arterial temperature *T*_*A*_ = 39.5°C (transient case).

**Figure 8:** Temperature distribution in the domain after tepid sponge treatment with initial fever or arterial temperature *T*_*A*_ = 41.0°C (transient case).

**Figure 9:** Comparison of temperature distribution in the domain before and after tepid sponge treatment with initial fever or arterial temperature *T*_*A*_ = 38.0°C (steady-state case).

**Figure 10:** Comparison of temperature distribution in the domain before and after tepid sponge treatment with initial fever or arterial temperature *T*_*A*_ = 41.0°C (transient case).

**Table 1:** Numerical computation of the temperature distribution *T*_*i*,*j*,*k*_ (°C) in the domain during tepid sponge treatment with fever or arterial temperature *T*_*A*_ = 38.0°C (steady-state case).

*i*	*j*	*k*	*T*_*i*,*j*,*k*_	*i*	*j*	*k*	*T*_*i*,*j*,*k*_	*i*	*j*	*k*	*T*_*i*,*j*,*k*_	*i*	*j*	*k*	*T*_*i*,*j*,*k*_
0	0	0	8.53												
0	1	0	9.72	0	-1	0	9.72	0	0	1	9.87	0	0	-1	9.87
0	1	1	11.17	0	-1	1	11.17	0	1	-1	11.21	0	-1	-1	11.21
1	0	0	10.89												
1	1	0	12.51	1	-1	0	12.51	1	0	1	12.58	1	0	-1	12.58
1	1	1	13.48	1	-1	1	13.48	1	1	-1	13.53	1	-1	-1	13.53
1	2	0	15.03	1	-2	0	15.03	1	0	2	15.06	1	0	-2	15.06
1	2	1	16.32	1	-2	1	16.32	1	2	-1	16.29	1	-2	-1	16.29
1	2	2	18.25	1	-2	2	18.25	1	2	-2	18.27	1	-2	-2	18.27
2	0	0	18.02												
2	1	0	20.35	2	-1	0	20.35	2	0	1	20.38	2	0	-1	20.38
2	1	1	22.79	2	-1	1	22.79	2	1	-1	22.76	2	-1	-1	22.76
2	2	0	24.00	2	-2	0	24.00	2	0	2	24.03	2	0	-2	24.03
2	2	1	27.65	2	-2	1	27.65	2	2	-1	27.68	2	-2	-1	27.68
2	2	2	28.78	2	-2	2	28.78	2	2	-2	28.81	2	-2	-2	28.81
3	0	0	29.11												
3	1	0	31.34	3	-1	0	31.34	3	0	1	31.37	3	0	-1	31.37
3	1	1	32.68	3	-1	1	32.68	3	1	-1	32.71	3	-1	-1	32.71
3	2	0	34.03	3	-2	0	34.03	3	0	2	34.05	3	0	-2	34.05
3	2	1	35.21	3	-2	1	35.21	3	2	-1	35.24	3	-2	-1	35.24
3	2	2	37.03	3	-2	2	37.03	3	2	-2	37.35	3	-2	-2	37.35

**Table 2:** Numerical computation of the temperature distribution *T*_*i*,*j*,*k*_ (°C) in the domain during tepid sponge treatment with fever or arterial temperature *T*_*A*_ = 39.5°C (steady-state case).

*i*	*j*	*k*	*T*_*i*,*j*,*k*_	*i*	*j*	*k*	*T*_*i*,*j*,*k*_	*i*	*j*	*k*	*T*_*i*,*j*,*k*_	*i*	*j*	*k*	*T*_*i*,*j*,*k*_
0	0	0	9.13												
0	1	0	9.94	0	-1	0	9.94	0	0	1	9.98	0	0	-1	9.98
0	1	1	11.23	0	-1	1	11.23	0	1	-1	11.28	0	-1	-1	11.28
1	0	0	11.09												
1	1	0	12.71	1	-1	0	12.71	1	0	1	12.68	1	0	-1	12.68
1	1	1	13.74	1	-1	1	13.74	1	1	-1	13.77	1	-1	-1	13.77
1	2	0	15.58	1	-2	0	15.58	1	0	2	15.61	1	0	-2	15.61
1	2	1	16.54	1	-2	1	16.54	1	2	-1	16.51	1	-2	-1	16.51
1	2	2	18.44	1	-2	2	18.44	1	2	-2	18.73	1	-2	-2	18.73
2	0	0	18.92												
2	1	0	20.85	2	-1	0	20.85	2	0	1	20.83	2	0	-1	20.83
2	1	1	23.07	2	-1	1	23.07	2	1	-1	23.10	2	-1	-1	23.10
2	2	0	24.26	2	-2	0	24.26	2	0	2	24.63	2	0	-2	24.63
2	2	1	28.15	2	-2	1	28.15	2	2	-1	28.18	2	-2	-1	28.18
2	2	2	29.08	2	-2	2	29.08	2	2	-2	29.01	2	-2	-2	29.01
3	0	0	29.20												
3	1	0	31.94	3	-1	0	31.94	3	0	1	31.97	3	0	-1	31.97
3	1	1	32.75	3	-1	1	32.75	3	1	-1	33.87	3	-1	-1	33.87
3	2	0	35.23	3	-2	0	35.23	3	0	2	35.25	3	0	-2	35.25
3	2	1	36.11	3	-2	1	36.11	3	2	-1	36.13	3	-2	-1	36.13
3	2	2	37.82	3	-2	2	37.82	3	2	-2	37.85	3	-2	-2	37.85

**Table 3:** Numerical computation of the temperature distribution *T*_*i*,*j*,*k*_ (°C) in the domain during tepid sponge treatment with fever or arterial temperature *T*_*A*_ = 41.0°C (steady-state case).

*i*	*j*	*k*	*T*_*i*,*j*,*k*_	*i*	*j*	*k*	*T*_*i*,*j*,*k*_	*i*	*j*	*k*	*T*_*i*,*j*,*k*_	*i*	*j*	*k*	*T*_*i*,*j*,*k*_
0	0	0	9.72												
0	1	0	10.12	0	-1	0	10.12	0	0	1	10.17	0	0	-1	10.17
0	1	1	11.41	0	-1	1	11.41	0	1	-1	11.62	0	-1	-1	11.62
1	0	0	12.01												
1	1	0	13.16	1	-1	0	13.16	1	0	1	13.19	1	0	-1	13.19
1	1	1	13.93	1	-1	1	13.93	1	1	-1	13.96	1	-1	-1	13.96
1	2	0	15.88	1	-2	0	15.88	1	0	2	15.91	1	0	-2	15.91
1	2	1	16.67	1	-2	1	16.67	1	2	-1	16.71	1	-2	-1	16.71
1	2	2	18.76	1	-2	2	18.76	1	2	-2	18.80	1	-2	-2	18.80
2	0	0	19.09												
2	1	0	20.98	2	-1	0	20.98	2	0	1	21.04	2	0	-1	21.04
2	1	1	23.24	2	-1	1	23.24	2	1	-1	23.22	2	-1	-1	23.22
2	2	0	24.34	2	-2	0	24.34	2	0	2	24.76	2	0	-2	24.76
2	2	1	28.24	2	-2	1	28.24	2	2	-1	28.41	2	-2	-1	28.41
2	2	2	29.53	2	-2	2	29.53	2	2	-2	29.71	2	-2	-2	29.71
3	0	0	29.82												
3	1	0	32.14	3	-1	0	32.14	3	0	1	32.19	3	0	-1	31.19
3	1	1	33.06	3	-1	1	33.06	3	1	-1	34.02	3	-1	-1	34.02
3	2	0	35.63	3	-2	0	35.63	3	0	2	35.59	3	0	-2	35.59
3	2	1	36.23	3	-2	1	36.23	3	2	-1	36.21	3	-2	-1	36.21
3	2	2	37.95	3	-2	2	37.95	3	2	-2	37.97	3	-2	-2	37.97

**Table 4:** Numerical computation of the temperature distribution *T*_*i*,*j*,*k*_ (°C) in the domain during tepid sponge treatment with fever or arterial temperature *T*_*A*_ = 38.0°C (transient case).

*i*	*j*	*k*	*T*_*i*,*j*,*k*_			*i*	*j*	*k*	*T*_*i*,*j*,*k*_		
			*t* = 2 min	*t* = 4 min	*t* = 6 min				*t* = 2 min	*t* = 4 min	*t* = 6 min
0	0	0	14.21	12.43	11.65	0	1	0	14.63	13.31	12.90
0	-1	0	14.63	13.31	12.90	0	0	1	14.94	14.43	14.05
0	0	-1	14.94	14.43	14.05	0	1	1	15.36	14.82	14.28
0	1	-1	15.36	14.82	14.28	1	0	0	15.83	15.43	15.20
1	1	0	16.66	16.35	15.92	1	-1	0	16.66	16.35	15.92
1	0	1	17.23	16.84	15.31	1	0	-1	17.23	16.84	15.31
1	1	1	17.84	17.54	15.15	1	-1	1	17.84	17.54	15.15
1	1	-1	18.27	17.93	17.24	1	-1	-1	18.27	17.93	17.24
1	2	0	18.75	18.34	17.93	1	-2	0	18.75	18.34	17.93
1	0	2	19.32	18.73	18.22	1	0	-2	19.32	18.73	18.23
1	2	1	19.92	19.65	19.31	1	-2	1	19.92	19.65	19.31
1	2	-1	20.47	20.03	19.74	1	-2	-1	20.47	20.03	19.74
1	2	2	21.05	20.64	20.23	1	-2	2	21.05	20.64	20.23
1	2	-2	21.82	21.52	21.12	1	-2	-2	21.82	21.52	21.12
2	0	0	22.73	22.37	21.84	2	1	0	23.13	22.77	22.25
2	-1	0	23.13	22.77	22.25	2	0	1	23.81	23.44	22.83
2	0	-1	23.81	23.44	22.83	2	1	1	24.58	24.13	23.65
2	-1	1	24.58	24.13	23.65	2	1	-1	24.95	24.64	24.27
2	-1	-1	24.95	24.64	24.27	2	2	0	25.05	24.73	24.18
2	-2	0	25.05	24.73	24.18	2	0	2	25.64	25.34	24.72
2	0	-2	25.64	25.34	24.72	2	2	1	26.19	25.87	25.36
2	-2	1	26.19	25.87	25.36	2	2	-1	26.72	26.41	25.93
2	-2	-1	26.72	26.41	25.93	2	2	2	27.14	26.83	26.33
2	-2	2	27.14	26.83	26.33	2	2	-2	27.66	27.28	26.67
2	-2	-2	27.66	27.28	26.67	3	0	0	29.25	28.85	28.10
3	1	0	29.83	29.34	28.95	3	-1	0	29.83	29.34	28.95
3	0	1	30.45	30.04	29.43	3	0	-1	30.45	30.04	29.43
3	1	1	30.82	30.44	29.96	3	-1	1	30.82	30.44	29.96
3	1	-1	31.53	30.93	30.15	3	-1	-1	31.53	30.93	30.15
3	2	0	31.91	31.22	30.35	3	-2	0	31.91	31.22	30.35
3	0	2	32.66	32.14	31.45	3	0	-2	32.66	32.14	31.45
3	2	1	33.14	32.74	32.16	3	-2	1	33.14	32.74	32.16
3	2	-1	33.83	33.26	32.68	3	-2	-1	33.73	33.26	32.68
3	2	2	34.92	34.62	34.44	3	-2	2	34.92	34.62	34.44
3	2	-2	36.16	35.96	35.83	3	-2	-2	36.16	35.96	35.83

**Table 5:** Numerical computation of the temperature distribution *T*_*i*,*j*,*k*_ (°C) in the domain during tepid sponge treatment with fever or arterial temperature *T*_*A*_ = 39.5°C (transient case).

*i*	*j*	*k*	*T*_*i*,*j*,*k*_			*i*	*j*	*k*	*T*_*i*,*j*,*k*_		
			*t* = 2 min	*t* = 4 min	*t* = 6 min				*t* = 2 min	*t* = 4 min	*t* = 6 min
0	0	0	14.44	12.53	11.94	0	1	0	14.83	13.52	13.31
0	-1	0	14.83	13.52	13.31	0	0	1	15.13	14.66	14.29
0	0	-1	15.13	14.66	14.29	0	1	1	15.54	15.03	14.57
0	1	-1	15.54	15.03	14.57	1	0	0	16.04	15.72	15.37
1	1	0	16.84	16.53	16.15	1	-1	0	16.84	16.53	16.15
1	0	1	17.53	17.05	15.64	1	0	-1	17.53	17.05	15.64
1	1	1	18.16	17.77	15.36	1	-1	1	18.16	17.77	15.36
1	1	-1	18.43	18.15	17.54	1	-1	-1	18.43	18.15	17.54
1	2	0	18.93	18.53	18.26	1	-2	0	18.93	18.53	18.26
1	0	2	19.55	18.94	18.55	1	0	-2	19.55	18.94	18.55
1	2	1	20.17	19.81	19.53	1	-2	1	20.17	19.81	19.53
1	2	-1	20.62	20.22	19.91	1	-2	-1	20.62	20.22	19.91
1	2	2	21.33	20.92	20.55	1	-2	2	21.33	20.92	20.55
1	2	-2	22.07	21.77	21.35	1	-2	-2	22.07	21.77	21.35
2	0	0	22.96	22.55	21.97	2	1	0	23.34	22.93	22.57
2	-1	0	23.34	22.93	22.57	2	0	1	24.04	23.64	23.13
2	0	-1	24.04	23.64	23.13	2	1	1	24.82	24.33	23.88
2	-1	1	24.82	24.33	23.88	2	1	-1	25.15	24.94	24.59
2	-1	-1	25.15	24.94	24.59	2	2	0	25.23	24.96	24.33
2	-2	0	25.23	24.96	24.33	2	0	2	25.91	25.63	24.92
2	0	-2	25.91	25.63	24.92	2	2	1	26.35	26.04	25.55
2	-2	1	26.35	26.04	25.55	2	2	-1	26.91	26.62	26.16
2	-2	-1	26.91	26.62	26.16	2	2	2	27.33	27.05	26.68
2	-2	2	27.33	27.05	26.68	2	2	-2	27.92	27.55	26.98
2	-2	-2	27.92	27.55	26.98	3	0	0	29.33	29.07	28.34
3	1	0	30.16	29.66	29.14	3	-1	0	30.16	29.66	29.14
3	0	1	30.63	30.23	29.65	3	0	-1	30.63	30.23	29.65
3	1	1	31.07	30.67	30.15	3	-1	1	31.07	30.67	30.15
3	1	-1	31.73	31.13	30.44	3	-1	-1	31.73	31.13	30.44
3	2	0	32.18	31.59	30.68	3	-2	0	32.18	31.59	30.68
3	0	2	32.84	32.33	31.77	3	0	-2	32.84	32.33	31.77
3	2	1	33.35	32.95	32.39	3	-2	1	33.35	32.95	32.39
3	2	-1	34.04	33.44	32.88	3	-2	-1	34.04	33.44	32.88
3	2	2	35.13	34.81	34.72	3	-2	2	35.13	34.81	34.72
3	2	-2	36.34	36.17	36.05	3	-2	-2	36.34	36.17	36.05

**Table 6:** Numerical computation of the temperature distribution *T*_*i*,*j*,*k*_ (°C) in the domain during tepid sponge treatment with fever or arterial temperature *T*_*A*_ = 41.0°C (transient case).

*i*	*j*	*k*	*T*_*i*,*j*,*k*_			*i*	*j*	*k*	*T*_*i*,*j*,*k*_		
			*t* = 2 min	*t* = 4 min	*t* = 6 min				*t* = 2 min	*t* = 4 min	*t* = 6 min
0	0	0	14.62	12.83	12.15	0	1	0	14.92	13.77	13.33
0	-1	0	14.92	13.77	13.33	0	0	1	15.33	14.98	14.55
0	0	-1	15.33	14.98	14.55	0	1	1	15.77	15.26	14.77
0	1	-1	15.77	15.26	14.77	1	0	0	16.24	15.96	15.66
1	1	0	17.05	16.77	16.33	1	-1	0	17.05	16.77	16.33
1	0	1	17.76	17.33	15.94	1	0	-1	17.76	17.33	15.94
1	1	1	18.34	17.95	15.66	1	-1	1	18.34	17.95	15.66
1	1	-1	18.77	18.45	17.86	1	-1	-1	18.77	18.45	17.86
1	2	0	19.15	18.74	18.59	1	-2	0	19.15	18.74	18.59
1	0	2	19.73	19.23	18.86	1	0	-2	19.73	19.23	18.86
1	2	1	20.34	20.15	19.87	1	-2	1	20.34	20.15	19.87
1	2	-1	20.92	20.42	20.14	1	-2	-1	20.92	20.42	20.14
1	2	2	21.63	21.13	20.86	1	-2	2	21.63	21.13	20.86
1	2	-2	22.27	21.96	21.66	1	-2	-2	22.27	21.96	21.66
2	0	0	23.14	22.77	21.96	2	1	0	23.55	23.11	22.76
2	-1	0	23.55	23.11	22.76	2	0	1	24.25	23.85	23.34
2	0	-1	24.25	23.85	23.34	2	1	1	25.16	24.56	24.18
2	-1	1	25.16	24.56	24.18	2	1	-1	25.44	25.17	24.83
2	-1	-1	25.44	25.17	24.83	2	2	0	25.71	25.35	24.96
2	-2	0	25.71	25.35	24.96	2	0	2	26.13	25.91	25.15
2	0	-2	26.13	25.91	25.15	2	2	1	26.67	26.26	25.77
2	-2	1	26.67	26.26	25.77	2	2	-1	27.28	26.98	26.44
2	-2	-1	27.28	26.98	26.44	2	2	2	27.66	27.25	26.94
2	-2	2	27.66	27.25	26.94	2	2	-2	28.14	27.83	27.27
2	-2	-2	28.14	27.83	27.27	3	0	0	29.66	29.27	28.67
3	1	0	30.45	29.97	29.37	3	-1	0	30.45	29.97	29.37
3	0	1	30.93	30.53	29.96	3	0	-1	30.93	30.53	29.96
3	1	1	31.26	30.85	30.45	3	-1	1	31.26	30.85	30.45
3	1	-1	31.97	31.53	30.84	3	-1	-1	31.97	31.53	30.84
3	2	0	32.45	31.86	30.94	3	-2	0	32.45	31.86	30.94
3	0	2	33.14	32.66	32.05	3	0	-2	33.14	32.66	32.05
3	2	1	33.66	33.15	32.66	3	-2	1	33.66	33.15	32.66
3	2	-1	34.27	33.86	33.15	3	-2	-1	34.27	33.86	33.15
3	2	2	35.49	35.08	34.98	3	-2	2	35.49	35.08	34.98
3	2	-2	36.72	36.52	36.43	3	-2	-2	36.72	36.52	36.43

**Table 7:** Numerical values of the parameters.

S. no.	Property	Region	Num. value	Unit
01	Thermal cond.	Scalp	3.42 × 10^−1^	W/mK
		Skull	6.51 × 10^−1^	W/mK
		CSF	2.17 × 10^−1^	W/mK

02	Specific heat cap.	Scalp	3.6 × 10^3^	J/kgK
		Skull	1.59 × 10^3^	J/kgK
		CSF	2.36 × 10^3^	J/kgK
		Blood	4.01 × 10^3^	J/kgK

03	Density	Scalp	1.07 × 10^3^	kg/m^3^
		Skull	1.52 × 10^3^	kg/m^3^
		CSF	0.88 × 10^3^	kg/m^3^

04	Metab. heat gen.	Scalp (outer)	0	W/m^3^
		Scalp (inner)	1.8 × 10^3^	W/m^3^
		Skull	0	W/m^3^
		CSF	0.3 × 10^3^	W/m^3^

05	Blood perf. rate	Scalp	6.06 × 10^−3^	kgm^−3^s^−1^

06	Heat tran. coef.	Scalp	6.4 × 10^−1^	W/m^2^K

## Data Availability

No data has been used in this paper. The tables are numerical calculations and can be calculated by the reader himself with the help of equations and numerical values as given by Table 7.
